The article "Effect of High-Dose Vitamin D3 Intake on Ambulation, Muscular Pain and Bone Mineral Density in a Woman with Multiple Sclerosis: A 10-Year Longitudinal Case Report" was published in 2012. Journal: Int J Mol Sci.

# Effect of High-Dose Vitamin D3 Intake on Ambulation, Muscular Pain and Bone Mineral Density in a Woman with Multiple Sclerosis: A 10-Year Longitudinal Case Report

**DOI:** 10.3390/ijms131013461

**Published:** 2012-10-19

**Authors:** Barbara M. van Amerongen, François Feron

**Affiliations:** 1 Department of Molecular Cell Biology and Immunology, VU University Medical Center, 1017 MB Amsterdam, The Netherlands; 2 Department of Cariology Endodontology Pedodontology, Academic Centre for Dentistry, 1081 LA Amsterdam, Amsterdam, The Netherlands; 3 Aix Marseille Université, Centre National de la Recherche Scientifique (CNRS), NICN, UMR 7259, 13015, Marseille, France; E-Mail: francois.feron@univ-amu.fr

**Keywords:** vitamin D3, multiple sclerosis, ambulation, muscular pain, bone mineral density, 25(OH)D, PTH, 1,25(OH)2D, malabsorption, coeliac disease

## Abstract

Mounting evidence correlate vitamin D3 (cholecalciferol) supplementation or higher serum levels of vitamin D (25(OH)D) with a lower risk of developing multiple sclerosis (MS), reduced relapse rate, slower progression or fewer new brain lesions. We present here the case of a woman who was diagnosed with MS in 1990. From 1980 to 2000, her ability to walk decreased from ~20 to 1 km per day. Since January 2001, a vitamin D3 supplement was ingested daily. The starting dose was 20 mcg (800 IU)/day and escalated to 100 mcg (4000 IU)/day in September 2004 and then to 150 mcg (6000 IU)/day in December 2005. Vitamin D3 intake reduced muscular pain and improved ambulation from 1 (February 2000) to 14 km/day (February 2008). Vitamin D intake over 10 years caused no adverse effects: no hypercalcaemia, nephrolithiasis or hypercalciuria were observed. Bowel problems in MS may need to be addressed as they can cause malabsorption including calcium, which may increase serum PTH and 1,25(OH)2D levels, as well as bone loss. We suggest that periodic assessment of vitamin D3, calcium and magnesium intake, bowel problems and the measurement of serum 25(OH)D, PTH, Ca levels, UCa/Cr and bone health become part of the integral management of persons with MS.

## 1. Introduction

Vitamin D metabolism influences many tissues as most cells have vitamin D receptors [1], including immune and neural cells (for reviews, [2–4]). Mounting evidence correlate sun exposure, vitamin D3 (cholecalciferol) intake or higher serum levels of vitamin D (25(OH)D) with a lower risk of developing multiple sclerosis (MS), reduced relapse rate, slower progression of MS or lower development of new lesions on brain magnetic resonance imaging (MRI) [5–15], even in paediatric-onset MS [16].

One of these observational studies found that no relapse occurred when serum levels of 25(OH)D were above 85 nmol/L (34 ng/mL) or when serum levels of intact parathyroid hormone (iPTH) were below 2.2 pmol/L (20 ng/L), which corresponds to 30% of the corresponding upper reference limit (%URL) [11]. An Australian study reported that a 10 nmol/L increase in the vitamin D level may reduce the risk of a relapse up to 12%; the data implied that increasing serum 25(OH)D levels by 50 nmol/L could more than halve the risk of a relapse [17].

High serum levels of 25(OH)D may also halt the progression of the disease as a strong association was found between lower serum levels of 25(OH)D and higher disability Expanded Disability Status Scale score (EDSS > 3) [6,12]. Conversely, higher circulating levels of 25(OH)D were associated with a lower EDSS score [13]. An association between 25(OH)D levels and a decline in MRI brain lesions and brain atrophy has also been reported [14,15].

In early treatment studies, dietary supplementation with vitamin D and other nutrients had been found to decrease relapse rate in two small groups of young MS patients [18,19]. Supplementation of 1000 IU vitamin D3 per day for six months (vitamin D3, *n* = 17; placebo, *n* = 19) induced elevated circulating TGF-β1 levels, a potential indicator of vitamin D action in MS [20]. A seven-month safety study in 12 patients, supplemented with 2800 to 28,000 IU vitamin D3 per week, reported a decline in the number of demyelinating plaques but without any observed symptom improvement [21]. More recently, MS patients (vitamin D3, *n* = 23; placebo, *n* = 22), treated with escalating doses of vitamin D3 over 12 months, displayed, apart from a reduced relapse rate, a persistent reduction in T cell proliferation [22,23]. Three months supplementation with a daily dose of 20,000 IU vitamin D3 (*n* = 15) resulted in a more anti-inflammatory cytokine profile [24].

A monthly intra muscular injection of 300,000 IU vitamin D3 in Iranian MS patients (vitamin D3, *n* = 26; placebo, *n* = 33) for six months showed no significant differences in clinical or MRI outcomes, however increased anti-inflammatory cytokines IL-10 and TGF-β levels were found [25].

Many of the vitamin D and MS studies to date are observational in nature rather than randomized placebo controlled trials. However, these early clinical trials provide a learning curve. For example, the two recent, double blind, phase IV randomized placebo controlled trials with weekly delivery of 20,000 IU vitamin D3 conducted by neurologists in Norway and Finland [26,27] assessed clinical MS-related outcomes, including relapse rate, EDSS and duration of a 25 foot walk (T25FW) but the size of the cohort (around 35 individuals in each arm) did not allow definitive conclusions to be drawn.

Some of the currently enrolling randomized (placebo) controlled trials, when sufficiently powered, may be able to provide meaningful results. Merck Serono SA started recruiting patients for a two and a three-arm, randomized, double-blind, placebo controlled, multicenter, phase II study to evaluate the efficacy of vitamin D3 (Vigantol^®^ Oil) as add-on therapy in subjects with relapsing remitting (RR)MS receiving treatment with Rebif^®^, namely the CHOLINE trial (*n* = 250) [28] and the SOLAR trial (*n* = 358) [29,30]. In another two-year long trial by Johns Hopkins and UCSF, patients (*n* = 172) will be assigned to low dose (600 IU/day) versus high-dose (5000 IU/day) of vitamin D3 as an add-on therapy to glatiramer acetate (Copaxone) [31].

The first vitamin D clinical trial for the prevention of MS in patients with Clinically Isolated Syndrome (CIS) will take place in Australia and New Zealand and is due to start in 2012 and will run for four years, up to 2016. It is a placebo controlled, trial (*n* = 290) that will test three dosage levels of daily vitamin D3 supplements (1,000, 5,000 and 10,000 IU) against placebo tablets (PrevANZ Vitamin D MS prevention trial, not yet registered).

Nonetheless, results will not become available for several years and it remains of interest to accumulate individual evidence on the role of vitamin D in MS.

### 1.1. Endpoints

MS is an inflammatory disease of the central nervous system, provoking demyelination and axonal degeneration. It generally induces a partial paralysis and around 50% of MS patients become at least dependent on a walking aid after 15 years of disease while only 10% are free of major disability after 20–25 years [32].

It has been long known that vitamin D protects against muscle weakness [33]. Low vitamin D levels have been associated with increased body sway, changes in gait, difficulties in rising from a chair and inability to ascend stairs [34]. In rats, vitamin D regulates intracellular phosphate in muscle [35], improves muscle anabolism [36] and induces a fast-to-slow fiber type transition of the Tibialis anterior muscle, after a peroneal nerve section [37]. In humans, delivery of a vitamin D analogue, for 3 to 6 months, to older patients with osteoporosis increased the percentage and area of type-2 (fast-twitch) muscle fibers [38]. A low dose of vitamin D2, given over a period of two years to 48 elderly hemiplegic women who were vitamin D-deficient, augmented the relative number and size of type II muscle fibers and improved muscle strength [39]. Finally, treatment of vitamin D deficiency with vitamin D3 and calcium increased lower limb muscle strength, independently of regular physical activity, in institutionalized older people [40].

It is well established that inadequate intake of vitamin D3 (and calcium) leads to reduced calcium absorption, chronic secondary hyperparathyroidism, higher bone remodeling rates and increased bone loss [41,42]. Causes of secondary hyperparathyroidism in women after menopause are low calcium nutrition or malabsorption, decreased renal function and low estrogen status [43].

Data suggest a significantly increased prevalence of bone loss in patients with MS compared to age-matched controls [44–48]. Patients (*n* = 2501) with MS often have multiple risk factors for osteoporotic fractures including impaired mobility (66%), falls in the last 12 months (55.2%), family history of osteoporosis (41.5%), sedentary life style (32.2%), low bone mass (27.2%), fracture (24.9%) and steroid use (5.6%) [49]. Low bone mass at early stages of disease in MS patients has been described [50]. MS may be a cause of secondary osteoporosis as both diseases share aetiological and pathogenic factors [51].

For all these reasons, we have focused our attention on the clinically meaningful outcome measures: ambulation (walking distance expressed in km/day) and muscular pain (painkillers yes/no), and on the surrogate outcome measures: Bone Mineral Density (BMD) [51], serum levels of 25(OH)D > 85 nmol/L [11,27], PTH < 2.2 pmol/L (20 ng/L) or < 30 %URL [11,27], and the urinary calcium to creatinine ratio UCa/Cr > 1.0 [52].

### 1.2. Biographical Data

A Caucasian woman, born in January 1950, living in the Netherlands (latitude 52°N), with a normal body mass index (BMI) of 20.2 (1990) was diagnosed with MS in 1990 (first symptoms in 1975), at the age of 40. The subject started taking vitamin D3 supplements in 2001, 26 years after the first symptoms of MS and 11 years after the diagnosis of MS. Her medical history revealed a diagnosis of idiopathic thrombocytopenic purpura (ITP) (Werlhof) in 1974, which was treated with prednisone until the platelet count was found to be within the normal range (NR) in 1977. However, in 1978, ITP reappeared and lasted several months. In Spring 1975, the first symptoms of MS emerged. Tingling sensations (paresthesia) in the left hand and tongue, followed in 1979 by symptoms of pain in the right leg and lack of coordination in the left. In 1992, a second opinion confirmed the diagnosis of MS. A brain MRI was taken in March 1990 and December 2004. The brain MRI in 1990 showed multiple T2-hyperintense white matter lesions in the peri-ventricular area, the corpus callosum and the medulla oblongata. The MRI in 2004 showed no new T2 lesions and no enhancement after contrast administration. Cerebrospinal fluid (CSF) was not analyzed. No vitamin deficiencies were identified or excluded. The Kurtzke EDSS score [53] was carefully assessed under standardized conditions by well-trained medical doctors [54,55]. The EDSS score was 3 in 1999 and 3 in 2012. Whilst the type of MS (disease course) was never specifically stated, according to the EDSS by definition this patient has benign MS and no disease modifying treatment (DMT) was ever prescribed.

In 2011 the subject was clinically diagnosed with Coeliac Disease (CD) (first symptoms in childhood). Eating Wiener schnitzel caused Gastrointestinal (GI) symptoms. During puberty, drinking milk, eating cheese or eggs caused severe headaches. After puberty, drinking beer caused restless legs. Subject simply stopped eating Wiener schnitzel, drinking milk and beer.

GI symptoms became more apparent during time spent in Singapore. Bread and fried foods containing soy sauce (which has wheat as an ingredient) caused bloating and constipation. The subject visited a gastroenterologist for the first time in August 1998. The subject smoked until the age of 42. In 1997, the subject had to resign dental practice due to fatigue.

During the period of vitamin D intake (2001 onwards), the medication history revealed no disease modifying treatment (DMT), no cod liver oil or other medications that affect vitamin D and calcium metabolism, except for estradiol. Estradiol was taken from 1992 until menopause in 2002, to regulate the menstrual cycle. In 2009, eight years after the beginning of vitamin D and calcium supplementation, the subject was diagnosed with osteopenia. At present, the subject uses no stick or wheelchair.

Details of the methods used, including Study Design (4.1.), Vitamin D3 and Calcium Supplementation (4.2.), Exercise (4.3.), Blood sampling (4.4.), and Bone Mineral Density (4.5.) are provided in the Experimental Section.

## 2. Results

### 2.1. Biochemical Assessment

All biochemical measurements were within their corresponding NR, except for 1,25(OH)2D on four out of nine occasions (Table 1).

#### 2.1.1. Serum 25(OH)D

A dose of 20 mcg (800 IU)/day of vitamin D3 (January 2001) resulted in a serum 25(OH)D level of 102 nmol/L after 10 months (November 2001) but, 34 months later, the 25(OH)D level declined to 84 nmol/L (October 2004). The ingested dose was then increased from 20 to 100 mcg (4000 IU)/day of vitamin D3 (September 2004). This resulted in a 25(OH)D level of 102 nmol/L after 12 months (September 2005). The dose was increased again this time from 100 to 150 mcg (6000 IU)/day of vitamin D3 (December 2005). This dose stabilized the 25(OH)D level above 135 nmol/L (Table 1/Figure 1a). Although there were rises and falls in the 25OHD level throughout the 10 year period, since 2001, the patient’s 25OHD level was always within a “safe” physiological range of 75–200 nmol/L [52].

#### 2.1.2. Serum PTH

The first PTH measurement showed a high-normal value, namely 72 %URL (November 2001). At that time, a daily supplement of 800 IU vitamin D3 and 240 mg calcium was ingested. After increasing vitamin D3 intake by 500% from 20 to 100 mcg (800 to 4000 IU)/day, the PTH level did not fall but rose 9% (from 75 to 82 %URL) after 12 months. After increasing vitamin D3 intake for the second time by 50%, from 100 to 150 mcg (4000 to 6000 IU)/day, PTH fell 20% (from 82 to 64 %URL) after 12 months.

From January 2001, a daily dietary supplement of 240 mg elemental calcium was ingested. As from March to July 2009, the subject was supplemented four times a day with 333 mg elemental calcium (including magnesium, zinc and copper). The serum level of PTH declined by 32% (from 79 to 54 %URL) after six months. In 2010, PTH increased to 93 %URL, as no calcium supplements were taken (Table 1 and Figure 1b).

#### 2.1.3. Serum 1,25(OH)2D

The NR of 1,25(OH)2D is 50–180 pmol/L. Serum 1,25(OH)2D fluctuated between 55 and 255 pmol/L. On four out of nine occasions 1,25(OH)2D reached levels above 180 pmol/L, the URL.

From March to July 2009, the subject was supplemented four times a day with 333 mg elemental calcium (including magnesium, zinc and copper). The serum level of 1,25(OH)2D declined by 46% (from 119 to 55 pmol/L) (Table 1 and Figure 1b).

### 2.2. Ambulation

Subject always liked walking, even when she could not walk very fast or for a long distance. Over the years, the subject performed several trips that lasted more than one-day. On the basis of those trips, it has been estimated how many kilometers the subject was able to walk in a single day (Figure 2).

In 1983–1985, the walking distance was ~20 km/day but, in 1985, walking companions started to complain about the slowness of the subject. At the end of the day, the subject was the only one suffering from severe calf muscle pain. Just before the diagnosis of MS (1990), the subject was still able to walk ~16 km/day. In 1995, subject’s walking ability dropped to ~5 km/day. Around 2000, the subject only managed to walk ~1 km/day. At that time, she did not feel confident to go out on her own.

In 2005, after four years of vitamin D3 and calcium supplementation, subject’s walking ability improved to ~5 km/day and by 21 February 2008, the subject was able to walk ~14 km in 4 h (2 h one way, and after a 2 h lunch, 2 h return) in one day without calf muscle pain.

In March 2012, the subject walked 5 km in 60 min and the subject was able to run a short distance, *i.e.* for catching a bus. Subject’s balance had improved and she could stand without feeling pain at night time. In addition, it must be highlighted that no relapse was diagnosed by a neurologist during the vitamin D supplementation period.

### 2.3. Muscular Pain

Vitamin D3 supplementation has reduced the pain to a level that allowed the subject to stop using a painkiller (Paracetamol). Even after a long walk, the subject no longer suffers from muscular pain, whether calf muscle pain or nocturnal leg cramps.

### 2.4. Bone Mineral Density

BMD was determined four times with a dual-energy X-ray absorptiometer (DEXA), at Year 9 (1999), 19 (2009), 20 (2010) and 21 (2011) post-MS diagnosis (Table 2). The first BMD measurement at the lumbar spine (LS) was normal. Ten years later, data at the LS and left proximal femur (LPF) indicated osteopenia (−2.5 < *T*-score < −1.0). From 2009 to 2011 (10 and 12 years after the first BMD), BMD at the PF decreased by 6.3% (0.05 g/cm^2^) from 0.788 to 0.738 g/cm^2^. The most recent *Z*-score at the LS and LPF was −0.6 and −0.8, respectively.

### 2.5. Adverse Events

Adverse events including hypercalcaemia, nephrolithiasis or fracture, were not observed. Serum calcium levels remained within the NR. In January 2009, a scan with a sonographer revealed no renal calculus (kidney stones) after eight years of vitamin D3 supplementation. Additionally, no hypercalciuria (UCa/Cr > 1.0) was observed 2.21/3.6 = 0.61 (July 2011) (endpoint).

## 3. Discussion

An earlier case report describing the effects of high-dose vitamin D3 on biochemical parameters has been published but that report did not mention ambulation, muscular pain or BMD of the MS patient [56]. In this current report, a dose of vitamin D3 up to 150 mcg (6000 IU)/day administered for 10 years resulted in a serum level of 25(OH)D above 135 nmol/L (endpoint) but did not result in a serum PTH level of less than 30 %URL (endpoint), despite the high serum level of 25(OH)D.

### 3.1. 25(OH)D, PTH and 1,25(OH)2D Levels

After augmenting the daily vitamin D3 intake from 800 to 4000 IU (20 to 100 mcg), the serum level of 25(OH)D increased from 84 (October 2004) to 102 nmol/L (September 2005), a dose-response of 5.6 nmol/L after 12 months for every 1000 IU/day of vitamin D3 added. After the second augmentation, from 4000 to 6000 IU (100 to 150 mcg)/day, the serum level of 25(OH)D increased from 102 (September 2005) to 138 nmol/L (October 2006), a dose-response of 18 nmol/L after 12 months for every 1000 IU/day of vitamin D3 added.

Comparably, a weekly dose of 20,000 IU (500 mcg) of vitamin D3 and 500 mg elemental calcium, ingested for 96 weeks, plateaued the median vitamin D level to 123 nmol/L, which corresponds to a dose-response of 25 nmol/L for every 1000 IU/day of vitamin D3 supplemented [48].

The dose-responses of the subject after one year—respectively, 5.6 nmol/L and 18 nmol/L for every 1000 IU/day of vitamin D3—were below the reported dose-response of ~25 nmol/L for every 1000 IU/day of vitamin D3 supplemented [48]. This indicates that absorption of vitamin D3 was not adequate. Malabsorption such as that found in CD may compromise the absorption of vitamin D3 [43].

It is important to state here that it requires eight months to attain a final plateau—a steady state—in the serum 25(OH)D concentration from the start of a new or additional vitamin D3 dose [57].

Malabsorption is only one of the many variables that affect vitamin D levels. Causes of vitamin D deficiency in general include reduced skin synthesis, decreased bioavailability (malabsorption and obesity), increased catabolism, acquired and heritable disorders (rickets) (for a review, [58]).

In dogs, the LD50 (the lethal dose which kills 50% of the animals) for cholecalciferol is a one-time dose of over 3,000,000 IU/kg [59], whereas in the case of human beings, the oral delivery of cholecalciferol, at doses exceeding 500 IU/kg/day (37,500 IU/day for a person weighing 75 kg) given up to two months, was found to be safe [60]. No imbalance of the phosphocalcic homeostasis and no hypercalcaemia or hypercalciuria was noticed in people treated with an average dose of 14,000 IU/day of cholecalciferol over one year [22]. However, it has been observed that delivery of 500,000 IU vitamin D3 to elderly community-dwelling women, as a one-time annual maintenance dose, resulted in increased risks of falls and fractures [61]. A safer way would have been to provide cholecalciferol at the weekly rate of 100,000 IU, for 5 consecutive weeks, and then start the regular maintenance dose after one week [57].

A negative correlation between 25(OH)D and PTH level illustrating a tight feedback regulation resulting in a stable 1,25(OH)2D and Ca concentration is usually reported [62]. However, over a period of 10 years, an inverse relationship between 25(OH)D and PTH (*r* = −0.02) was only observed once at the increase of vitamin D3 supplementation or when the subject was supplemented with calcium 4 times per day. This observation is against the odds for this being chance alone. In a three month trial with a cholecalciferol intake of 20,000 IU per day without calcium supplementation, a decrease in PTH was observed after 1.5 months. In vitamin D treated patients, median PTH at baseline was 4.6 (range 1.9–10.5) pmol/L and 2.8 (range 1.7–6.7) pmol/L, 1.5 months later [24]. Conversely, a one year study with a seven times lower cholecalciferol intake of 20,000 per week, with a mean (SD) calcium intake of 1150 (502) mg per day, delivers a different outcome. In this double blind, placebo controlled, randomized trial, PTH suppression was not obtained in either treatment arm, after 12 months [27]. An earlier Finish study reported winter hypercalcaemia and a blunted PTH response in MS patients compared to controls. The possibility was raised that the endocrine circuitry regulating serum calcium is altered in MS patients either as a cause or a consequence of their disease [11].

PTH measuremets are important to prevent relapses and bone resorption in MS. Relapses in multiple sclerosis occur when intact PTH serum levels are > 30 %URL. Noteworthy, only 38% of patients in remission have intact PTH levels ≤ 30 %URL [11]. Continuous secretion of excess PTH causes bone resorption [63].

Increased 25(OH)D levels did not affect circulating 1,25(OH)2D concentrations when calcium (1200 mg/day) was prescribed [23]. Conversely, in a three month trial with a cholecalciferol intake of 20,000 IU per day without calcium supplementation, median circulating 1,25(OH)2D levels rose from 146 to 202 (range 151–535) pmol/L and stabilized after four weeks [24]. Of note, no calcium will be delivered to patients enrolled in the two-year long SOLAR follow-up trial [30].

Calcium intake remains an important issue. Ionized serum calcium levels are critical for the correct functioning of multiple vital cellular processes. Accordingly, the regulation of calcium homeostasis is directed at maintaining serum calcium levels within a narrow physiological range. Briefly, hypocalcemia leads to increased PTH secretion, which stimulates renal calcium reabsorption and bone resorption. PTH also enhances production of 1,25(OH)2D, which activates the vitamin D receptor (VDR), leading to an increased calcium absorption in the intestine and bone resorption in the skeleton [64].

A reduced PTH level has been observed when (1) vitamin D3 was ingested [65], (2) 25(OH)D levels were equal or above 100 nmol/L (40 ng/mL) [66], (3) short term 1,25(OH)2D therapy (1 mcg at bedtime for 8 days) was provided to elderly subjects [67], (4) individuals had a calcium intake of 2400 mg/day over a three year period [68] and (5) oral supplementation with high frequency calcium intake (up to four times per day) was delivered [69]. Magnesium citrate (1830 mg/day) intake for 30 days also reduced the PTH level as magnesium regulates PTH secretion [70]. Conversely, low dietary calcium intake or calcium malabsorption in CD, leads to higher PTH levels (secondary hyperparathyroidism), higher 1,25(OH)2D levels and a reduced half life of 25(OH)D, as well as bone loss [43,71,72]. It can therefore be surmised that the comorbid CD diagnosed in the subject has counterbalanced the vitamin D effect on 25(OH)D, PTH and 1,25(OH)2D levels.

### 3.2. Calcium and Magnesium Supplementation

Surprisingly, no mention of additional magnesium intake was reported in the above mentioned clinical trials. To our knowledge and according to a vast review of available data, only one study indicates that a group of MS patients (*n* = 16) was treated with dietary supplements containing vitamin D3 (125 mcg (5000 IU)/day), calcium (16 mg/kg/day), and magnesium (10 mg/kg/day) [18].

Calcium in combination with magnesium, zinc and copper is necessary for the formation of bone and teeth and for normal nerve and muscle function. Magnesium deficiency has been associated with a number of clinical disorders including osteoporosis [73]. Low magnesium intake may influence MS disease progression as well [74].

As shown in Table 1, the measured serum total magnesium (Mg^t^) was always sufficient. However, low levels of the physiologically active form of magnesium (Mg^2+^) indicates hypomagnesemia more accurately [75].

### 3.3. Ambulation

The subject was evaluated every year by a neurologist. The EDSS score was evaluated on two occasions, in 1999 and in 2012. The EDSS defines “fully ambulatory” as “at least 500 meters of ambulation”, either “unrestricted” or “restricted (EDSS ≥ 2)”. As a result “walking distance per day (km/day)” was used as a clinically meaningful outcome measure for MS disease progression. The reverse of MS symptoms was related in time to highly ingested quantities of vitamin D3 and the improvement in ambulation preceded the GFD.

The mechanisms underlying such a recovery can be multiple. It is now well established that vitamin D plays an immuno-modulatory role [2]. This neurosteroid hormone is involved in many autoimmune diseases [76], including MS [77]. As a general rule, hypovitaminosis D is a risk factor for MS [78] and it has been shown, in an animal model of MS, that the severity of the symptoms is reduced when vitamin D is provided during early life [79].

In addition, accumulating evidence indicate that vitamin D is a potent neurotrophic agent [78] which promotes axon regeneration [37,80] and reduces demyelination [81]. Moreover, the muscle is now recognised as a target for vitamin D. Vitamin D increases the percentage of type-2 (fast-twitch) muscle fibers [38,39] and increases lower limb muscle strength in institutionalized older people [40]. These findings, in combination with studies on athletes, have led to the conclusion that vitamin D may improve physical performance [82].

Interestingly, an iterative process could be at play. Indeed, the recovery described in this report could also be the consequence of the regular training performed by the subject. Arguably, vitamin D3 and calcium intake led to physical recovery, which enabled the subject to exercise. The subject executed Alexander Technique lessons and exercises with a Swiss Ball, a procedure used in physical therapy for neurodevelopmental treatment [83,84]. This activity is known to enhance motor control.

### 3.4. Muscular Pain

Pain is a common symptom in patients with MS, paracetamol was used at a daily dose of 2–4 tablets (500 mg) at night. The subject simply noticed that she stopped buying and using painkillers. “Painkillers per day (yes/no)” was used as a clinically meaningful outcome measure for MS muscular pain. At this stage, very little is known about the role of vitamin D on chronic pain. There is evidence that vitamin D supplementation can relieve musculoskeletal pain [85–87].

Furthermore, pain sensitive dorsal root ganglia (DRG) neurons express the major vitamin D machinery metabolites (nuclear receptor and limiting enzyme), suggesting that they respond to vitamin D [88] and a recent study has shown that vitamin D deficiency likely contributes to muscular hypersensitivity and pain [89]. However, the mechanisms remain obscure and new studies are required to fully assess the role of vitamin D on algesia and allodynia.

### 3.5. Bone Mineral Density

A normal first BMD measurement at the lumbar spine (LS), nine years post-MS diagnosis, is not in line with the findings of low bone mass at early stages of disease [50]. Therefore it comes as a surprise that the subject, supplemented with a high dose of vitamin D3, was diagnosed with osteopenia, eight years after the start of vitamin D supplementation. It can be argued that the condition could have been worse without vitamin D intake. Additional explanations can be proposed.

First, the endpoint of a serum PTH level of less than 30%URL has not been achieved, despite supplementation with 150 mcg (6000 IU/day) of vitamin D3, resulting in a serum level of 25(OH)D above 135 nmol/L (54 ng/mL). Arguably, lower serum levels of PTH may be desirable in alleviating symptoms of MS and preventing bone loss.

Second, the subject was poorly compliant for calcium intake, as the intake of calcium supplements increased GI symptoms. In clinical studies, calcium supplementation caused GI side effects in 16% and in 22% of the MS patients, which lead to discontinuation of the supplement [22,26]. In both studies, the cause of the GI symptoms was not reported. Dietary calcium tolerance is an important issue since calcium malabsorption increases vitamin D turnover due to secondary hyperparathyroidism, as well as bone loss [43].

Third, GI symptoms seem to be a common condition in MS since 55% of 17,030 MS patients report bowel problems, defined as “any difficulty in passing faeces including constipation, bowel incontinence, and diarrhoea” [90]. As reported by Katz and Weinerman, “Gastrointestinal disease is often overlooked or simply forgotten as a cause of osteoporosis” [91].

Fourth, in July 2011, thirteen years after her first visit to a gastroenterologist, the subject’s physician confirmed the diagnosis of CD [92]. CD is a major cause of intestinal malabsorption, including calcium [72]. Calcium malabsorption stimulates the secretion of PTH causing hyperparathyroidism. Untreated CD is characterized by high levels of PTH and high levels of 1,25(OH)2D. Furthermore, an inverse relationship between PTH and bone density or 1,25(OH)2D and bone density in coeliac patients has been reported [72,93]. After being diagnosed with CD a strict gluten (and lactose and coffee) free diet (GFD) was established. This diet resolved bloating and constipation. Since then, the subject has resumed calcium intake.

### 3.6. Limitations of the Study

Smoking is clearly a confounding factor. It is associated with increased MS susceptibility. Available evidence associates cigarette smoking with a greater chance of developing progressive disease and accruing more rapid disability [94]. However, the subject stopped smoking nine years before vitamin D intake.

At least two other confounding factors—hormone replacement and physical therapy—can be listed. It has been demonstrated that pregnancy-associated hormones alter immune responses and MS pathogenesis (for a recent review, [95]) and it can be hypothesized that delivery of estradiol has affected the course of MS for this patient. However, it must be mentioned that estrogen replacement was delivered early on and the concomitance with vitamin D3 treatment lasted only a year. Similarly, a meta-analysis suggests that exercise therapy can be beneficial for patients with MS not experiencing an exacerbation [96]. Alexander technique lessons corrected the gait disturbance and allowed the subject to walk longer distances. Interestingly, the exercise therapy prescribed by the neurologist of the subject to improve her gait did not improve her ambulation in the years before vitamin D3 intake.

One can wonder about the reliability of the MS diagnosis. No CSF has ever been analyzed and only two EDSS scores were recorded. However, neurologist and MRI data are unambiguous. Multiple white matter lesions matching MS were observed and the neurologist who examined the subject in June 2012, for a clinical trial entitled “Mechanisms of disability in MS patients with long disease duration”, confirmed the diagnosis of benign MS.

The current case report would have benefited from more regular EDSS assessments since it is a universally recognized outcome measure. However, the first symptoms of MS occurred in 1975, 15 years prior to the diagnosis. Naturally no EDSS scores were available for those 15 years. However, because the subject enjoyed walking holidays with her friends but found she could not keep up with them, she began monitoring her ambulation since 1980 so that she might predetermine the distance she would be able to walk and plan future trips without being left behind. For the past 30 years she has been recording her ambulation in km/day, under the control of her friends.

It also must be highlighted that EDSS defines “fully ambulatory” as “at least 500 meters of ambulation”, either “unrestricted” or “restricted (EDSS ≥ 2)”. The subject’s ambulation was restricted, but she had always been able to walk 500 meters and, as a consequence, the EDSS is not appropriate to detect improvement in medium and long distance walking. This is illustrated by the fact that the EDSS score has not changed in 13 years: 3 in 1999 and 3 in 2012. This in itself is a positive outcome in MS.

Likewise, a meta-analysis on the effectiveness of exercise therapy for MS reported the outcome measures Timed Walk 6, 10 or 50 meters and failed to find any effect on EDSS and concludes: “There is an urgent need for consensus on a core set of outcome measures to be used in exercise trials” [96].

A *n* of 1 case study has limited value, when compared with a properly run randomized controlled trial. However, it must be highlighted that most of the previous clinical trials include biases, are underpowered or not randomized. In the end, they are not necessarily much more informative than detailed case studies, such as the current one. Conversely, well known neurologists have started to prescribe vitamin D to their patients and an increasing number of MS individuals are self-medicating with (high) doses of vitamin D. These patients need to be monitored. Currently, assessments of high vitamin D intake are not performed appropriately. The current manuscript may provide valuable information on how to monitor MS patients, at least until the results of clinical trials and evidence-based guidelines are published.

### 3.7. Data Collection

It must be pointed out that the data were not always collected in the same hospital. Furthermore, the assay method used within the same hospital changed over time. Generally speaking, the hospitals did not provide information on the assays used for the biochemical assessments, including 25(OH)D and PTH serum concentrations. PTH was analyzed by different assay methods and their reference ranges were dissimilar. For this reason the NR of PTH was not provided. Expressing the PTH values as a percentage of the corresponding URL, provided by the hospitals, enabled comparison.

Two out of four BMD measurements were performed on the same scanner. Hospitals did not provide data on the calibration of the scanner.

### 3.8. One Person and Three Autoimmune Diseases

Epidemiological studies have found a prevalence of ITP in MS patients about 25-fold higher than in the general population [97,98]. The benefit of adequate 25(OH)D levels in ITP has been reported [99]. The prevalence of CD is 1%–2% worldwide in the general population but 11% in MS patients [100]. An overlap in the genetic risk loci for CD and MS has been reported [101,102]. Similarly, a positive association between ITP and CD, irrespective of which disease came first, has also been reported [103]. Altogether, these data suggest common mechanisms that lead to the development of autoimmune diseases. Gluten sensitivity can cause a range of neurological manifestations (for a review, [104]). CD alone can cause neurological symptoms that can mimic those of MS [105,106]. To exclude CD in MS patients should become a standard procedure.

## 4. Experimental Section

### 4.1. Study Design

This was a 10-year longitudinal case study.

### 4.2. Vitamin D3 and Calcium Supplementation

From 1992 up till now, during wintertime in Netherlands, the subject spent at least one month in Singapore (latitude 1°N). The notion that the incidence of MS was lower around the Equator prompted the subject to spend time in Singapore during winter, when the UV index was too low to induce a satisfactory production of vitamin D3 in the Netherlands. On average a Dutch person ingests 200 IU/day vitamin D3 from food [107].

The subject started ingesting a vitamin D3 supplement in January 2001, at the dose of 800 IU (20 mcg)/day, together with a daily dietary supplement of 240 mg elemental calcium (1,000 mg calcium citrate powder). Ten months later (November 2001), the vitamin D level was measured for the first time and was 102 nmol/L. In September 2004, the vitamin D3 dose prescribed by her neurologist, increased from 800 to 4000 IU (100 mcg)/day. As the serum level of 25(OH)D did not increase enough in response to the higher vitamin D3 intake and the serum level of PTH did not decrease, the vitamin D3 dosage was raised further in December 2005, this time from 4000 to 6000 IU (150 mcg)/day (Table 1/Figure 1a).

Dietary calcium supplements are not recommended in the Netherlands, as the Dutch Health Council (Gezondheidsraad) is of the opinion that Dutch food contains enough calcium (milk) [107]. As the subject hardly ever drank milk, a daily dietary supplement of 240 mg elemental calcium (1000 mg calcium citrate powder) was ingested.

In January 2009, the subject was diagnosed with osteopenia. From March to July 2009, she started ingesting a different calcium supplement. One serving size (three tablets) contained 1 g of elemental calcium (as Calcium Carbonate) and 400 mg of magnesium (as Magnesium Oxide). Each serving also supplied the added benefit of 15 mg of zinc (as Zinc Oxide) and 1 mg of copper. Instead of taking one tablet three times a day, the subject took one tablet four times a day, thus increasing the serving size by 4/3 (Figure 1b). After July 2009, compliance to calcium intake became poor because of GI symptoms.

### 4.3. Exercise

The exercise therapy prescribed by her neurologist since 1990 to improve her gait prior to vitamin D3 intake did not improve her ambulation.

Vitamin D3 and calcium supplementation enabled the subject to exercise again. In 2007, she resumed Alexander Technique lessons, once prescribed by her neurologist in 1976. Alexander Technique is a technique of body re-education and coordination. It aims to develop lifelong skills for self-care that help people recognize, understand and avoid poor habits affecting postural tone and neuromuscular coordination [83]. These lessons improved her gait and enabled her to walk longer distances. Since 2008, the subject exercises, once a week for one hour, in a small group with a professional instructor. In addition, once every 2 weeks, the subject has an individual lesson on the Swiss Ball [84]. The subject walks outdoors, every day, for a period ranging from 12 to 60 min. To measure walking distance and speed, an electronic pedometer (DIGI-WALKER Yamax SW 650) was used.

### 4.4. Blood Sampling

Serum levels of 25(OH)D, 1,25(OH)2D, PTH, calcium, creatinine, phosphate, ALP, albumin, and magnesium were measured at yearly intervals over the 2001–2011 period (Table 1). The selection of biochemical indices of bone metabolism was made on the basis of a previous paper [13]. Blood samples were obtained after at least 8 h of fasting. Ionized calcium was not assessed, as the albumin levels were normal.

### 4.5. Bone Mineral Density

Osteoporosis is diagnosed when BMD is less than or equal to 2.5 or more standard deviations below peak bone mass (*i.e.* the *T*-score is −2.5 or above) while osteopenia is defined as a *T*-score between −1 and −2.5. The *Z*-score is the number of standard deviations a patient’s BMD differs from the average BMD for their age, sex, and ethnicity.

## 5. Conclusions

The current case report provides interesting information on the therapeutic benefit of long-term administration of cholecalciferol in one patient. This case also highlights the need to consider the co-occurrence of other autoimmune diseases such as CD in MS [100]. The report demonstrates that moderately high doses of vitamin D3 over a prolonged period are safe. This finding is also relevant for MS patients without CD. Supplementation with vitamin D3 may improve ambulation and reduce muscular pain. Randomized placebo controlled trials are necessary to validate these effects of vitamin D supplementation in MS. High vitamin D levels may reduce, though not necessarily prevent, bone loss in MS. Intake of high vitamin D3, calcium and magnesium should be monitored by regular assessments of (i) bowel problems (ii) serum 25(OH)D, PTH and Ca levels (iii) urinary calcium to creatinine ratio (UCa/Cr) and (iv) BMD. The vitamin-D related serum levels should preferably be assessed once a year in summer when 25(OH)D levels are high in order to treat existing vitamin D deficiency or to prevent serum 25(OH)D levels from declining in winter. If vitamin D levels are checked in winter and the level is deficient, lower than 75 nmol/L, it is simply too late to correct the deficiency because it takes months to synthesize the enzymes necessary for an optimal vitamin D metabolism [57]. Optimal serum 25(OH)D levels are those that are both high in the physiologic range, and stable throughout the year [57].

## Figures and Tables

**Figure 1:** Dose escalation of vitamin D3 (mcg/day) and calcium (cg/day) supplementation, serum levels of 25(OH)D in nmol/L (endpoint 25(OH)D level > 85 nmol/L), PTH in % upper reference limit (URL) (endpoint PTH level < 30 %URL) and 1,25(OH)2D in pmol/L (NR 1,25(OH)2D 50–180 pmol/L). (**a**) Vitamin D3 supplementation (mcg/day), serum levels of 25(OH)D in nmol/L, serum levels of PTH in %URL and serum levels of 1,25(OH)2D in pmol/L; (**b**) Calcium supplementation (cg/day), serum levels of 25(OH)D in nmol/L, serum levels of PTH in %URL and serum levels of 1,25(OH)2D in pmol/L.

**Figure 2:** Ambulation, walking distance expressed in km/day and vitamin D3 supplementation (mcg/day).

**Table 1:** Biochemical assessment (*n* = 1).

Date			5 December 2001	4 October 2004	29 September 2005	24 March 2006	5 October 2006	17 October 2007	28 January 2009	28 July 2009	23 June 2010	7 June 2011

Hospital			a	b	b	b	b	b	c	b	b	d

Blood test	Unit	NR										
25(OH)D	nmol/L	>50	102	84	102	84	138	142	145	201	204	135
1,25(OH)2D	pmol/L	50–180	147	164	**237**	**187**	172	119	nd	55	**213**	**255**
PTH	pmol/L	7.9	4.1	4.5	3.6	3.5	4.3	5.4	3.7	6.3	3.2	
PTH	%URL	< 30	72	75	82	66	64	63	79	54	93	72
Calcium	mmol/L	2.2–2.6	2.25	2.34	2.34	2.29	2.32	2.38	2.37	2.42	2.32	2.34
Magnesium	mmol/L	0.7–1.0	nd	0.9	0.8	0.8	0.9	0,8	nd	nd	0.9	0.8
Phosphate	mmol/L	0.7–1.4	0.87	1.20	1.10	1.00	1.00	1.00	1.30	nd	1.20	1.17
Creatinine	mmol/L	60–110	85	75	74	64	70	76	70	nd	73	67
Albumin	g/L	35–50	nd	40	41	39	40	38	42	nd	39	44
ALP	IU/L	40–120	65	79	74	79	80	63	nd	nd	73	47

a: VU University Medical Center, Amsterdam; b: BovenIJ Hospital, Amsterdam; c: Tan Tock Seng Hospital, Singapore; d: Onze Lieve VrouwenGasthuis, Amsterdam; ALP: Alkaline Phosphatase; NR: normal rang [13]; PTH was analysed by different assay methods. For this reason the NR of PTH is not provided. The PTH values are expressed as a percentage of the corresponding upper reference limit (%URL) provided by the hospitals; 1,25(OH)2D values out of the NR are in bold font; nd: no data.

**Table 2:** Bone Mineral Index and Bone Mineral Density for Lumbar Spine and Left Proximal Femur.

Date	Supplementation			Hospital	BMI	Location	BMD g/cm^2^	*T*-Score (SD)	*Z*-Score (SD)
	VD3 mcg/day	Ca mg/day	Mg mg/day						
1 January 1980	0	0	-	-	-	-	-	-	-
22 November 1999	0	0	-	a	21.6	LS	0.990	-0.5	nd
9 January 2001	20	240/1day	-	-	-	-	-	-	-
4 September 2004	100	240/1day	-	-	-	-	-	-	-
21 December 2005	150	240/1day	-	-	-	-	-	-	-
28 January 2009	150	240/1day	-	b	22.8	LS LPF	0.873 0.788	−1.6 −1.3	−0.2 −0.4
10 March 2009	150	333/4day	133/4day	-	-	-	-	-	-
27 July 2009	150	0	-	-	-	-	-	-	-
22 June 2010	150	0	-	c	20.8	LS L2 t/m 4 LPF	0.962 0.755	−2.0 −1.9	−0.7 −0.7
16 May 2011	150	0	-	c	20.5	LS L2 t/m 4 LPF	0.966 0.738	−2.0 −2.2	−0.6 −0.8
5 July 2011	150	145/4day	237/4day	-	-	-	-	-	-

a: VU University Medical Centre, Amsterdam; b: Tan Tock Seng Hospital, Singapore; c: Onze Lieve VrouwenGasthuis, Amsterdam; LS: Lumbar Spine; LPF: Left Proximal Femur.

## Abbreviations

ALP: alkaline phosphatase
BMD: bone mineral density
BMI: body mass index
CD: coeliac disease
EDSS: expanded disability status scale
GI: gastrointestinal
GFD: gluten free diet
ITP: idiopathic thrombocytopenic purpura
MS: multiple sclerosis
NR: normal range
RRMS: relapsing remitting MS
PTH: parathyroid hormone
URL: upper reference limit
%URL: as a % of the corresponding upper reference limit
